RETRACTED

# Multirobot Collaborative Pursuit Target Robot by Improved MADDPG

**DOI:** 10.1155/2022/4757394

**Published:** 2022-02-25

**Authors:** Xiao Zhou, Song Zhou, Xingang Mou, Yi He

**Affiliations:** ^1^School of Mechanical and Electronic Engineering, Wuhan University of Technology, Wuhan 430070, China; ^2^Intelligent Transport Systems Research Center, Wuhan University of Technology, Wuhan 430063, China

## Abstract

Policy formulation is one of the main problems in multirobot systems, especially in multirobot pursuit-evasion scenarios, where both sparse rewards and random environment changes bring great difficulties to find better strategy. Existing multirobot decision-making methods mostly use environmental rewards to promote robots to complete the target task that cannot achieve good results. This paper proposes a multirobot pursuit method based on improved multiagent deep deterministic policy gradient (MADDPG), which solves the problem of sparse rewards in multirobot pursuit-evasion scenarios by combining the intrinsic reward and the external environment. The state similarity module based on the threshold constraint is as a part of the intrinsic reward signal output by the intrinsic curiosity module, which is used to balance overexploration and insufficient exploration, so that the agent can use the intrinsic reward more effectively to learn better strategies. The simulation experiment results show that the proposed method can improve the reward value of robots and the success rate of the pursuit task significantly. The intuitive change is obviously reflected in the real-time distance between the pursuer and the escapee, the pursuer using the improved algorithm for training can get closer to the escapee more quickly, and the average following distance also decreases.

## 1. Introduction

The research of multirobot system has been widely applied in industrial manufacturing, medical health, military operations, and other fields. The multirobot system [1] first appeared in the 1970s, due to the demand of practical application is increasing, it is difficult for a single robot to handle a lot of complex tasks, researchers have gradually turned their attention to multirobot systems. Unlike single robot system, multiple robots can share information to learn better strategy to accomplish cooperative tasks. The learning mechanism in the multirobot system enables robots to acquire environmental perception, information memory, and behavioral decision-making abilities in the process of interacting with the environment.

The multirobot systems application is pursuit-evasion problem that is a typical problem in the study of multiagent cooperation and coordination strategies [2]. In essence, the pursuit-evasion problem is a multiagent cooperative decision problem. Robots study the optimal decision algorithm in multirobot system through the cooperative competition between the pursuers and the evaders. The methods to solve the problem of multirobot pursuit-evasion are mainly divided into the difference method and the combination method. The former converts the physical constraints of the robot into differential constraints and models and can only obtain local optimal solutions, but this method is widely used in solving the “simultaneous arrival” problem. [3]. The idea of latter method is to convert the pursuit problem into graph theory or dynamic programming problem and use greedy optimal return [4, 5], model predictive control [6], and other methods to learn the optimal strategy of the robot. Greedy algorithm [7, 8] is a typical combination method to fulfil the distance assignment task. This algorithm mainly realizes the allocation by minimizing the distance between the robot and the target. The application of this method is simple and extensive, but there will be a situation of allocation “deadlock.” Reference [9] uses the negotiation method [10] to redistribute the coincidentally assigned round-up points that effectively settle the problem of deadlock. Traditional methods usually require complex mathematical calculation process to solve the multirobot pursuit-evasion problem. With the development of artificial intelligence, more researchers adopt machine learning methods to seek optimal chasing strategies.

RETRACTED

Deep reinforcement learning (DRL) is a new machine learning method combining deep learning (DL) and reinforcement learning (RL). Compared with supervised and unsupervised learning, deep reinforcement learning combines the perceptual ability of deep learning with the decision-making ability of reinforcement learning [11] providing a solution to the complex and uncertain environment problems in multirobot systems [12, 13]. Volodymyr et al. first proposed deep Q-learning network (DQN) and obtained superhuman performance on Atari video games [14]. DQN is only applicable to discrete action space, and deep deterministic policy gradient (DDPG) is proposed to settle continuous action space issues [15]. Multiagent DDPG (MADDPG) is a multiagent policy gradient algorithm where agents learn a centralized critic based on the observation and actions of all agents [16, 17]. This method has already applied in the field of multirobot system. Kwak et al. [18] used reinforcement learning to train multirobot systems to obtain the optimal pursuit time. Li et al. [19] combined the data mining method of association rules with reinforcement learning and proposed a segmented reinforcement learning method, which solved the chase problem in the known environment. Liu et al. [20] used layered reinforcement learning to train the pursuit robot and designed an independent learning mechanism for the upper and lower stages [20] to balance the value function of different stages. The deep reinforcement learning method formulates an end-to-end strategy and is more targeted than traditional methods. However, the problem of inconsistent pursuit strategies in the phased training still exist. Additionally, the rewards of multirobot hunting scenes are sparse, and the algorithm stability performance is not satisfactory.

RETRACTED

This paper considers the pursuit-evasion problem and uses a deep reinforcement learning technique to solve this problem. The sparse rewards and excessive exploration affect the training process of the robot, resulting in the failure to complete the pursuit mission. This paper proposes an improved MADDPG multiagent decision-making algorithm via combining environmental rewards and intrinsic rewards. The purpose of this paper is to solve the problem of excessive exploration after adding intrinsic rewards and sparse environmental rewards in multirobot pursuit-evasion. This method adds a curiosity module based on state similarity to the robot's reward function, under the premise of ensuring that the pursuit task is completed, a greater cumulative return is obtained. In addition, a threshold for similarity constrains the amount of intrinsic reward to overcome the problem of overexploration. The idea of this method is to combine environmental rewards and intrinsic rewards to facilitate the robot to learn better policies. This idea is maybe a general idea for improving multiagent decision-making algorithms.

## 2. Multirobot Chase Model

### 2.1. Robot Motion Model

In the multirobot pursuit-evasion problem, this paper treats the individual robot as a particle, and the motion model of the robot is established in a two-dimensional plane. Both pursuers and evaders are randomly distributed in a 2D plane, and the dynamics model is the same for each robot. The information for each robot includes coordinate, velocity, direction, and detection radius, as shown in Figure 1. The kinematics model of the *i* th robot is expressed bywhere (*x*_*i*_, *y*_*i*_) represents the coordinate position of the *i*th robot, *r*_*i*_ is the radius of the sensing field of the *i*th robot, *θ*_*i*_ is the included angle between the heading and the horizontal direction of the robot, *v*_*i*_ represents the robot speed along the heading, *u*_*i*_ is the change rate of the heading angle of the *i*th robot, and *f*_0_ is the damping coefficient.


(1) $$\begin{array}{c} \left\{\begin{array}{c} x=x_{i},\\ y=y_{i},\\ r=r_{i},\\ v_{x_{i}}=v_{i}\cos\;\theta_{i},\\ v_{y_{i}}=v_{i}\sin\;\theta_{i},\\ \dot{\theta }=u_{i},\\ f=f_{0}. \end{array}\right. \end{array}$$

RETRACTED

### 2.2. Multirobot Cooperative Pursuit Problem

Multirobot cooperative pursuit is to study how to instruct a group of autonomous mobile robots (pursuers) to cooperate with each other to chase another group of mobile robots (evaders), which involves cooperation between pursers and confrontation between pursers and evaders [21]. Compared with single robot pursuit, the uncertainty of multirobot system environment and the diversity of information bring great difficulties to the pursuit task. The multirobot pursuit scenario is shown in Figure 2. The red circle represents the pursuer, the blue circle represents the evaders, and the gray area represents the obstacle. A collision occurs when the distance between the center of mass of the two objects is less than the sum of the radii of the two objects. The red robot needs to get as close as possible to the blue robot without collision between red robots to accomplish the pursuit task. The distance between red robot and blue robot is an indicator to measure the quality of the strategy. Red robot collides with blue robot is the best case but most case is that red robot follows blue robot keeping a certain distance.

There are some constraints in the multirobot pursuit-evasion scene. According to the robot motion model and multirobot pursuit process, the constraints are divided into control quantity constraint, initial state constraint, and distance constraint. Among them, the distance constraint including the obstacle constraint in the pursuit process of the robot and the safety distance constraint between the robots. The obstacle constraint requires no collision between robot and obstacle. Likewise, the safety distance constraint requires no collision between robots.

The control quantity constraint is reflected in the constraint on the change rate of the heading of each robot *u*_*i*_. *u*_*i*,max_ is the change rate of the maximum heading angle allowed by each robot, and the control quantity constraint of the *i*th robot is described as

(2) $$\begin{array}{c} \left|u_{i}\right|\leq u_{i,\text{max}}. \end{array}$$

The initial state includes the initial position and the initial heading angle, which are (*x*_0_, *y*_0_) and *θ*_0_, respectively. The initial constraint state corresponding to the *i*th robot is shown as

(3) $$\begin{array}{c} x_{i}\left(t_{1}\right)=x_{0},\\ y_{i}\left(t_{1}\right)=y_{0},\\ \theta_{i}\left(t_{1}\right)=\theta_{0}, \end{array}$$

where *x*_*i*_(*t*_1_), *y*_*i*_(*t*_1_), and *θ*_*i*_(*t*_1_) represent the coordinates and heading angle of the *i*th robot at the starting time *t*_1_.

RETRACTED

The distance constraint is embodied in the distance between robots and the distance between robots and obstacles. There are *N* obstacles as shown in the gray shadow part in Figure 2. In the process of cooperative pursuit, any pursuer must not collide with obstacles at any time and maintain a certain safe distance. Assuming that *D*_*i*_=[*x*_*i*_, *y*_*i*_]^*T*^, the obstacle constraint of the *i*th robot is expressed as

(4) $$\begin{array}{c} {\left|\left|D_{i}-D_{n}\right|\right|}_{2}\geq r_{n},\\ \forall i\in \left\{1,2,\ldots ,S\right\},\forall n\in \left\{1,2,\ldots ,N\right\}, \end{array}$$

where *n* is the number of the obstacle; *S* is the total number of pursuers; *N* is the total number of obstacles; *D*_*n*_ is the center coordinate of the *n*-th obstacle; and *r*_*n*_ is the maximum radius of the *n*th obstacle.

The safe distance of each pursuer is considered to avoid collision occurs. Pursuers need to meet the following constraints between each other described as

(5) $$\begin{array}{c} {\left|\left|D_{i}\left(t\right)-D_{j}\left(t\right)\right|\right|}_{2}\geq R_{s},\\ \forall t\in \left[t_{1},t_{f}\right],\forall i,j\in \left\{1,2,\ldots ,S\right\},i<j, \end{array}$$

where *R*_*s*_ is the safe distance between pursuers and *D*_*i*_(*t*) and *D*_*j*_(*t*) are the coordinates of *i*th and *j*th robot at time *t*.

## 3. Methods

### 3.1. Curiosity Module Based on State Similarity

Intrinsic curiosity module (ICM) [22] is a solution to the sparse reward and insufficient exploration motivation in multiagent environment. The error between the real state and the predicted state at the next moment is regarded as the intrinsic reward of agents in ICM to encourage agents to explore. According to the principle of intrinsic rewards, the larger the error between predicted state and real state, the more rewards agents obtain. Obeying this rule, supposing that the agent is exploring against real state direction at some point, it will always in wrong direction driven by abundant intrinsic reward that leads failure of pursuit task. Moreover, insufficient or excessive curiosity reward leads to unsatisfactory results [23]. Therefore, this paper adds a curiosity reward mechanism based on state similarity with threshold constraint on the basis of curiosity module. The degree of similarity between the predicted state and the real state represents the size of the prediction error, and the amount of intrinsic rewards to agents is effectively controlled by the constraint interval of similarity. When the similarity between the predicted state and the real state is below the lower threshold, agents cannot get internal excitation in order to prevent overexploration. In analogous cases, similarity exceeding higher threshold results in ignorance of intrinsic reward.

RETRACTED

The intrinsic curiosity module is composed of three parts of neural network, encoder module, forward state prediction network, and reverse action prediction network, as shown in Figure 3. The encoder is used for agent state feature extraction, and the forward module makes use of the current state ∅(*s*_*t*_) and the current action *a*_*t*_ to estimate the state of the next generation $\hat{\emptyset }\left(s_{t+1}\right)$. The inverse module employs a self-supervised style of predicting the current action by projecting forward the two ∅(*s*_*t*_) and ∅(*s*_*t*+1_) outputs of the network to predict action ${\hat{a}}_{t}$. The output of ICM is the two norm of $\hat{\emptyset }\left(s_{t+1}\right)$ and ∅(*s*_*t*+1_). Intrinsic rewards in this way do not take into account the problem of overexploration. Therefore, this method adds a similarity module to overcome this issue, as shown as Figure 3.

The state similarity module measures the degree of similarity between $\hat{\emptyset }\left(s_{t+1}\right)$ and ∅(*s*_*t*+1_) by the Pearson coefficient (as shown in equation (6)). At the same time, this method overcomes the under-reward and over-reward by the threshold constraint of similarity. The intrinsic rewards produced by state similarity module is described as equation (7), where *P* is the Pearson correlation coefficient between $\hat{\emptyset }\left(s_{t+1}\right)$ and ∅(*s*_*t*+1_) and *μ* is the reward coefficient. Agents only gain intrinsic reward when Pearson coefficient is between *low* and *high*, *low* is the lower boundary of *P*, while *high* is the upper boundary of *P*.

(6) $$\begin{array}{c} P\left(x,\;y\right)=\;\frac{E\left[\left(x_{i}-\bar{x}\right)\left(y_{i}-\bar{y}\right)\right]}{\sqrt{\sum_{i=1}^{n}{\left(x_{i}-\bar{x}\right)}^{2}}\sqrt{\sum_{i=1}^{n}{\left(y_{i}-\bar{y}\right)}^{2}}}, \end{array}$$

(7) $$\begin{array}{c} r_{t}^{i}=P*\mu \;\left(\text{low}<P<\text{high}\right). \end{array}$$

### 3.2. Improved MADDPG

Multiagent reinforcement learning algorithm is an effective method to settle the problem of multirobot pursuit-evasion. Each robot's decision is controlled by its own neural network, and the pursuers can complete the task of chasing fugitives through communication interaction and cooperative decision. MADDPG algorithm is improved on the basis of DDPG algorithm by Lowe ([16]) and applied to multiagent decision-making scenarios. Its core idea is to find the optimal global strategy by means of centralized training and distributed execution, which solves the problems of nonstationarity and the failure of experience replay method in multiagent environment. However, robots lack exploring motivation due to sparse rewards, which causes low rewards and model difficult to converge.

RETRACTED

This paper combines intrinsic reward and external environment reward as the agents' overall rewards via introducing the curiosity module based on state similarity into MADDPG. In this way, this method not only simulates the enthusiasm of the robot to study strategy but also prevents the excessive behavior. The model convergence speed and cumulative return value of the model are significantly improved using this method. Multiagent training is a process of searching for strategies that generate maximum total reward expectation and is described as shown in equation (8).

(8) $$\begin{array}{c} \underset{\theta_{p}}{\max}E_{\pi \left(s_{t};\theta_{p}\right)}\left[\sum_{t}r_{t}\right], \end{array}$$

where *θ*_*p*_ is the neural network parameter and *r*_*t*_ is the total reward value of the agent at time *T*. The total reward value consists of two parts, namely, the internal motivation is *r*_*t*_^*i*^ and the external environment motivation is *r*_*t*_^*e*^, as shown in equation (9). In general, the intrinsic motivation is 0. When the intrinsic curiosity module is added, the intelligence will take the similarity error between the predicted value and the actual value of the next state *s*_*t*+1_ as the intrinsic reward according to the current state *s*_*t*_ and the given action *a*_*t*_, as shown in

(9) $$\begin{array}{c} r_{t}=r_{t}^{i}+r_{t}^{e}. \end{array}$$

Improved MADDPG algorithm training framework adds an internal curiosity module on the basis of MADDPG, and its overall architecture is shown in Figure 4. As a whole, the actor-critic framework is still adopted [24, 25] Each agent is training by Actor network, Critic network, Target Actor network, and Target Critic network. The parameters of actor network and critic network are updated via gradient descent computing the overall loss. The parameters of the target network update via copying the parameters of the local network through soft update within a certain period of time.

This method adds a module named ICM, as shown in Figure 4. The inputs to this module are current real state *S*_*t*_, next real state *S*_*t*+1_, and current action *a*_*t*_ of each robot. The output is the intrinsic reward generating by state similarity module. The sum of intrinsic reward *r*_*t*_^*i*^ and external reward *r*_*t*_^*e*^ is put into replay buffer to update network. Through the optimized reward calculation method, the improved algorithm gives appropriate rewards to the robot resulting in better strategy that guides robots to catch up on the target robot faster and more accurately.

RETRACTED

### 3.3. Algorithm Process

The improved algorithm flow is shown in Table 1. Before training of agents, the replay buffer and exploration noise have been initialized, the network parameters of actor, critic, and the additional curiosity module also have been initialized. Every robot's state is reset at the begin of each episode, a quadruple *s*_*t*_, *a*_*t*_, *r*_*t*_, *s*_*t*_′ will update after each robot chooses an action and then is put into replay buffer, *s*_*t*_ and *s*_*t*_′ are robot's current state and next state, *a*_*t*_ is current action of robot, and *r*_*t*_ is the whole reward of robot. The value network and target network parameters will be updated by sampling in the replay buffer.

## 4. Design of the Multirobot Pursuit Strategy

### 4.1. State Space

For the multirobot pursuit-evasion scene, both the pursuer and the evaders are treated as particles, and the state space of the pursuit scene is divided into the pursuer and the evader.

The pursuer's state space includes the pursuer's centroid position *c*(*t*), the distance *d*(*t*) from other pursuer, the distance *l*(*t*) from the obstacle's centroid, the distance *w*(*t*) from the evader, the heading angle *φ*(*t*), and the heading speed *v*(*t*). The pursuer's state space at time *t* is defined as follows:

(10) $$\begin{array}{c} s_{r}\left(t\right)=\left[c\left(t\right),d\left(t\right),l\left(t\right),w\left(t\right),\varphi \left(t\right),v\left(t\right)\right]=\left[\begin{array}{c} \left(x,y\right),\left(d_{1},d_{2},\ldots ,d_{N}\right),\left(l_{1},l_{2},\ldots ,l_{M}\right),\left(w_{1},..,w_{K}\right),\\ \varphi ,\left(v_{x},v_{y}\right) \end{array}\right], \end{array}$$

where (*x*, *y*) is the pursuer's coordinate, (*d*_1_, *d*_2_,…, *d*_*N*_) is the distance between the current pursuer and peer pursuers, *N* is the number of peer pursuers, (*l*_1_, *l*_2_,…, *l*_*M*_) is the distance between the pursuer and the center of mass of the obstacle, *M* is the number of obstacles, (*w*_1_, .., *w*_*K*_) is the distance between the pursuer and the evader, *K* is the number of evaders, *φ* is the heading angle, and *v*_*x*_, *v*_*y*_ are the velocities along the *x* and *y* directions, respectively.

The state space of the evader includes the position *c*(*t*) of the center of mass of the evader, the distance *d*(*t*) between the evader and fellow evaders, the distance *l*(*t*) between the center of mass of the obstacle, the distance *w*(*t*) between the pursuer, the heading angle *φ*(*t*), and the heading speed *v*(*t*). The state space of the evader at time *t* is defined as follows:

(11) $$\begin{array}{c} s_{b}\left(t\right)=\left[c\left(t\right),d\left(t\right),l\left(t\right),w\left(t\right),\varphi \left(t\right),v\left(t\right)\right]=\left[\begin{array}{c} \left(x,y\right),\left(d_{1},d_{2},\ldots ,d_{K-1}\right),\left(l_{1},l_{2},\ldots ,l_{M}\right),\left(w_{1},..,w_{N+1}\right),\\ \varphi ,\left(v_{x},v_{y}\right) \end{array}\right]. \end{array}$$

RETRACTED

### 4.2. Action Space

This paper regards multirobot pursuit-evasion as a continuous process. Therefore, the action space is complex and continuous rather than simple and discrete. In accordance with the movement characteristics of the robot, the action space at time *t* is designed, as shown in

(12) $$\begin{array}{c} A\left(t\right)=\left\{\Delta \varphi ，\Delta v\right\}\\ =\left\{\varphi \left(t\right)+\mu t,v\left(t\right)+at\right\}, \end{array}$$

where Δ*φ* is the heading angle change value, *μ* is the angle change rate, Δ*v* is the heading velocity change value, and a is the acceleration. The movement process of the robot is mainly related to the speed and direction, angle change rate controls direction, and acceleration controls velocity.

### 4.3. Reward Function

With the design idea of improved MADDPG algorithm, the reward function is divided into two parts, including external environment reward and internal incentive reward.

In the multirobot pursuit-evasion scenario, pursuer is rewarded for catching up evaders. On the contrary, evaders who are caught are punished. However, sparse reward is not conducive to improving the comprehensive performance of the pursuer. Therefore, distance reward is also taken as an external reward in the design of reward function in this paper.

The relative position reward of the pursuer and the evader can be described, as shown in equation (13), *ω* is the relative distance reward coefficient, *M* is the number of pursuers, *N* is the number of evaders, *x*_predator_, *y*_predator_, *x*_prey_, *y*_prey_ are the *x* and *y* coordinates of the pursuer and the evader, respectively.

(13) $$\begin{array}{c} r_{t}^{e}=\omega *\sum_{i=1}^{M}\sum_{j=1}^{N}\left\|\left(x_{\text{predator}}^{i},y_{\text{prey}}^{i}\right)-\left(x_{\text{predator}}^{j},y_{\text{prey}}^{j}\right)\right\|. \end{array}$$

The reward of the pursuer for completing the pursuit task is described, as shown in equation (13). *δ* is the reward base value and the pursuer and the evader get negative reward.

(14) $$\begin{array}{c} r_{t}^{e}=\left\{\begin{array}{c} +\delta ,\;\text{if agent is predator,}\\ -\delta ,\;\text{if agent is prey.} \end{array}\right. \end{array}$$

As for intrinsic reward, it is designed to encourage robots to learn optimal strategy. This paper describes intrinsic reward as equation (15), *μ* is the reward coefficient and the intrinsic reward is generated by similarity error between the predicted state ${\hat{s}}_{t+1}$, and current state *s*_*t*+1_ at time *t*+1.

(15) $$\begin{array}{c} r_{t}^{i}=\mu *P\left({\hat{s}}_{t+1},s_{t+1}\right). \end{array}$$

The total reward *r*_*t*_ is the sum of external environment reward and internal incentive reward described as

(16) $$\begin{array}{c} r_{t}=r_{t}^{e}+r_{t}^{i}. \end{array}$$

RETRACTED

## 5. Simulation Experiment

### 5.1. Experimental Configuration

This paper adopts the hypothetical scenario in Figure 2 to complete a series of experiments, in which the pursuers cooperate to chase the evaders. The starting point of the task is when the pursuers start to move, and the end point is when they catch up with all the evaders. The simulation environment was redesigned on the basis of MPE environment and Python. OpenAI Gym reinforcement learning platform was adopted, and Pytorch deep learning framework was used to complete the simulation experiment of multirobot cooperative pursuit task.

The training of robots is a close-loop process, robots obtain environmental information by taking actions through strategy they have learned to update their own status information, then optimize pursuit-evasion strategy by means of the feedback information. The hyperparameters in the experiment are shown in Table 2. The whole training process iterates 2*∗*10^5^ times, each episode includes 100 steps. The critic network learning rate is slightly higher than actor network learning rate so that critic correctly guides actor. Discount factor represents the degree to which each training session is learned from the previous experience. The size of replay buffer and batch size depend speed of experience feedback. ΔT is the time interval for each simulation playback.

Different from deep learning, deep reinforcement learning has no data set. The agent obtains data from the simulation environment and uses the deep neural network for strategy optimization to train the model. Combined with the characteristics of deep reinforcement learning and the actual multirobot pursuit-evasion scenario, the following assumptions are made for the simulation environment:

1. To prevent the motivation generated by the internal curiosity module from keeping the robot exploring without stopping, this method limits environment boundaries and maximum stride length per turn.
2. All pursuers have exactly the same parameters, and they communicate with each other by share status information.
3. Considering the characteristics of deep reinforcement learning, the robot's range of activity is a two-dimensional infinite space. But the robot only moves within a certain range in practice, thereby this paper limits the multirobot pursuit scene to a two-dimensional finite space in that the robot is randomly initialized with coordinates between −1 and 1. Robots who are beyond the limited range are given certain punishment, and the environment is composed of *N* pursuers, *K* evaders, and *M* obstacles.

RETRACTED

### 5.2. Experimental Analysis

Deep reinforcement learning models usually judge algorithm performance from two aspects: convergence speed on the one hand and reward value after convergence on the other hand. In the experiment, the algorithm performance of MADDPG and the improved MADDPG algorithm in the multirobot pursuit-evasion problem are compared. Those methods including MADDPG, MADDPG with ICM, and improved MADDPG are tested in the 3VS1 scenario. The curve between the robot's average reward value and the number of iterations is drawn to evaluate the performance of algorithms, as shown in Figure 5. The reward value of the robot is the most intuitive manifestation of the performance of the algorithm. In the multirobot reinforcement learning training process, the average return value of the robot is calculated after each training episode to measure the quality of strategy and whether the algorithm has converged is judged by observing the training curve.

Figure 5 indicates that the overall average reward of the improved algorithm is significantly improved, and the method of adding state predicts error into intrinsic curiosity module accelerates the model convergence speed and has better convergence stability.

From the trend of the curves in Figure 5, the convergence value of the black curve (i.e., the MADDPG algorithm) is significantly lower than that of the other two curves. The red curve shows the trend of the reward value after adding the original curiosity module. The reward is increasing compared with MADDPG under the influence of increasing explore motivation via intrinsic reward generation by ICM. However, in the convergence stage, the curve oscillates greatly caused by excessive exploration. When the rules of giving intrinsic rewards are changed, the threshold of state similarity module limits intrinsic reward produced by ICM and guides the robot to explore rationally. Although the overall reward value is not greatly improved, the stability in the convergence stage is improved as shown by the blue curve.

In addition, in order to test the stability of the algorithm model, the trained model was tested in the 3VS1 scenario, and the average reward and task completion rate under 1000 tasks were counted. The results are shown in Figure 6 and Table 3.

RETRACTED

The test results shown in Figure 6 show that the improved MADDPG algorithm has significantly improved in both average reward value and task success rate. Taking task completion rate as a performance indicator, the improved algorithm has improved the success rate by 2–4 percentage points compared with the original algorithm.

Figure 6 shows the specific experimental data of the three algorithms in the form of a bar chart.  Figure 6(a) shows the average reward of the robot, and Figure 6(b) shows the success rate of the multirobot system under the three algorithms. Table 3 indicates that both reward and success rate are increasing and proves the effectiveness of the improved algorithm.

In the pursuit-evasion scenario of 3VS1, the distance between the pursuer and the evader is also an important indicator to measure the performance of the algorithm.  Figure 7 shows the track graph of a pursuit-evasion process and the real-time distance trend graph of the pursuer and the evader. The improved MADDPG algorithm enables the robot to follow the target more quickly and get closer to the target on average within the specified time. The statistical results are shown in Table 4.

The four pictures in Figure 7 intuitively show the robot's pursuit-evasion process, where Figures 7(a) and 7(c) are the trajectories of the robot tested using MADDPG and the improved algorithm. It is obvious that the improved algorithm drives more robots to approach the target robot, and their ability to follow the target is significantly improved. Figures 7(b) and 7(d) describe the real-time distance between the pursuer and the evader during the entire pursuit-evasion process. The average distance between the pursuer and the evader in a test is shown in Table 4. The improved algorithm can reduce the average distance between robot_1 and robot_2 and the target robot, which represents an improvement in the performance of robot hunting. Although robot_0 performs poorly, it does not affect the success of this pursuit task. One possible reason is that the robot sacrifices itself to provide other partners with richer information, thereby making other robots faster approach target.

## 6. Conclusion

To address the problem of changeable environment and sparse rewards in the process of multirobot pursuit-evasion, this paper proposes an intelligent multirobot pursuit-evasion method based on deep reinforcement learning. A multirobot pursuit-evasion model was built to describe motion model of robot and some constraints in the multirobot pursuit-evasion scene. The improved curiosity module with state similarity based on threshold constrain is introduced into the MADDPG algorithm to resolve sparse reward and unstable model caused by excessive exploration. The improved MADDPG algorithm is better applied to the multirobot pursuit-evasion scene by designing the state space, action space, and reward function of the agent. Comparing the improved MADDPG algorithm with the MADDPG algorithm, the results show that the improved algorithm can not only solve the problem of multirobot pursuit-evasion but also the average reward of the agent is obviously higher than the original algorithm.

RETRACTED

At present, the improved algorithm has better results for specific scenarios, the next step is to further optimize the algorithm so that it can play a better role in different scenarios.

## Figures and Tables

**Figure 1:** Robot motion model.

**Figure 2:** Schematic diagram of multirobot chase and escape scene.

**Figure 3:** Curiosity module based on state similarity.

**Figure 4:** Improved MADDPG algorithm framework.

**Figure 5:** Average reward value of simulation scenarios.

**Figure 6:** 1000-times test results. (a) Average reward. (b) Success rate.

**Figure 7:** Robot trajectory and real-time distance in the 3VS1 scenario. (a) Trajectory of the robot using MADDPG; (b) real-time distance between the pursuer and escaper using MADDPG; (c) trajectory of the robot using improved MA-DDPG; (d) real-time distance between the pursuer and esca-per using improved MADDPG.

**Table 1:** The multirobot collaborative pursuit strategy using improved-MADDPG.

(1). Initialize replay buffer *D* and motion exploration noise *ε*
(2). Initialize the EvalActor network and EevalCritic policy network for each robot
(3). Initialize the TargetActor network and TargetCritic network for each robot
(4). Initialize the ICM network for each robot
(5). For episode = 1 to MaxEpisode:
(6). Initialize the status of chase robot and escape robot *s*_*t*_
(7). For *t* = 1 to MaxStep:
(8). Each chaser and runner chooses the action *a*_*t*_
(9). Obtain *s*_*t*_, *a*_*t*_, *r*_*t*_^*e*^, *s*_*t*_′
(10). Calculate the intrinsic reward *r*_*t*_^*i*^ by *s*_*t*_ and *s*_*t*_′ similarity error *P*
(11). Update overall rewards *r*_*t*_=*r*_*t*_^*i*^+*r*_*t*_^*e*^
(12). Update current status *s*_*t*_′，push (*s*_*t*_, *a*_*t*_, *r*_*t*_, *s*_*t*_′) into replay buffer *D*
(13). For agent = 1 to *N*:
(14). Take *s* samples from the experience pool to form batch samples, and calculate union losses to update EvalCritic network parameter
(15). Soft update the TargetCritic network parameter
(16). End for
(17). Soft update TargetActor and TargetCritic network parameter
(18). End for
(19). End for

**Table 2:** The training hyperparameters.

Training parameter	Values

Max_steps	2*∗*10^5^
Maximum episode length step_len	100
Discount factor *γ*	0.96
Actor network learning rate *α*_*a*_	10^−4^
Critic network learning rate *α*_*c*_	10^−3^
Size of replay buffer *M*	10^6^
Batch size	256
Simulation time step Δ*T*	0.1 s

RETRACTED

**Table 3:** Average reward value and success rate.

Algorithm	Average	Success rate (%)	Improvement (%)

MADDPG	−15.3	84	—
ICM-MADDPG	−10.5	86.4	2.85
Ours	−9.1	87.2	3.81

**Table 4:** Average distance between the pursuer and evader in the 3VS1 scenario.

Algorithm	Average distance		
	robot_0	robot_1	robot_2

MADDPG	0.56	0.30	0.15
Ours	0.73	0.21	0.14

## Data Availability

No data set was used in this paper, and the data used in reinforcement learning were obtained by the agent from the simulation environment.
